# Explanatory Optimization of the Prediction Model for Building Energy Consumption

**DOI:** 10.1155/2022/9213975

**Published:** 2022-07-31

**Authors:** Huiyu Li, Hailong Dong

**Affiliations:** Department of Emergency Technology Management, Zhejiang College of Security Technology, Wenzhou 325006, China

## Abstract

Traditional prediction models, which are based on artificial neural networks (ANNs), consider the various factors affecting building energy consumption comprehensively. However, their explanatory power is not ideal in actual application, resulting in prediction errors of building energy consumption. Thus, this paper pursues the explanatory optimization of the prediction model for building energy consumption. First, the authors displayed the architecture of the prediction model for building energy consumption, which is based on the temporal pattern attention mechanism (TPAM), and explained the principle of predicting building energy consumption. Then, the input of the TPAM was illustrated, and the execution steps of the model were depicted. Based on feature importance and the Shapley additive explanations (SHAP) method, the explanatory power of the proposed prediction model was analyzed, from the perspective of the time series features of building energy consumption prediction. The proposed model was proved effective through experiments.

## 1. Introduction

With the rapid development of the economy, global energy consumption has increased year by year. Meanwhile, buildings become larger in scale, and better in grade, taking up a growing portion in global energy consumption. Therefore, it is practically significant to reduce the energy consumption, lower the emissions, and predict the energy consumption of large buildings [1–7]. For models with low data requirements, the trend of the time series for building energy consumption prediction can be obtained through simple statistical analysis of time nodes. Then, it is possible to make the final prediction of building energy consumption [8–17]. Traditional prediction models, which are based on artificial neural networks (ANNs), consider the various factors affecting building energy consumption comprehensively. However, their explanatory power is not ideal in actual application, resulting in prediction errors of building energy consumption. This significantly limits the applicable range of the models. As a result, it is necessary to develop models that can explain building energy consumption [18–21].

Nearly, 40% of global carbon emissions come from the building industry, which has a great potential for meeting the climate targets. Aiming to enhance building energy efficiency, the energy performance certificate requires accurate prediction of building energy performance. With the significant improvement of information and communication technology, the data-driven method has been introduced to study building energy performance and proved to boast a high computing efficiency and predictive performance. Nevertheless, most studies focus on predictive performance, without considering the potential of explaining artificial intelligence (AI). To fill up the gap, Wenninger et al. [6] designed the novel QLattice algorithm, which considers both predictive performance and the explanatory power. The algorithm was applied to forecast the annual energy-saving performance on a dataset containing 25,000 plus German residential buildings. Lei and Yin [22] improved the standard backpropagation (BP) neural network with the Levenberg–Marquardt (LM) algorithm and built an LMBP-based prediction model for the lighting energy consumption of high-rise buildings. The traditional prediction models for building energy consumption in shopping malls face limitations in the type and number of input variables. To overcome the limitations, Jing et al. [23] proposed a prediction model for building energy consumption in shopping malls based on the chaotic theory. The first step of the model is to compute the Lyapunov exponent of the energy consumption, which proves the chaotic nature of the energy consumption. As an important process in the sustainable building design, the evaluation of building energy-saving performance has a great impact on global energy reduction and environmental protection. Li et al. [24] developed an efficient way to evaluate building energy consumption. Their strategy integrates building information modeling (BIM), energy consumption simulation, and energy consumption prediction. The accurate prediction of building energy consumption is of great significance to the building energy management system. Nonetheless, building energy consumption is difficult to predict because the relevant data are often nonlinear and unsmooth. Karijadi and Chou [25] combined random forest (RF) and long short-term memory (LSTM) to predict building energy consumption, based on the complete ensemble empirical mode decomposition with adaptive noise (CEEMDAN).

Many studies have successfully predicted building energy consumption. Yet, most of them concentrate on improving prediction accuracy, summing up the key factors affecting building energy consumption, and the research trend of building energy prediction. The prediction effect of ensemble models depends on the basic learner and the ensemble strategy. It is impossible to demonstrate whether the model prediction is trustworthy or not. Thus, the prediction results often trigger many controversies. As a result, the building energy prediction models lack explanatory power. The model users in need of forecasting building energy consumption no longer trust the prediction results. In addition, the models are not frequently used in actual scenarios. Therefore, this paper pursues the explanatory optimization of the prediction model for building energy consumption.  Section 2 displays the architecture of the prediction model for building energy consumption, which is based on the temporal pattern attention mechanism (TPAM), and explains the principle of predicting building energy consumption.  Section 3 illustrates the input of the TPAM, and details the execution steps of the model.  Section 4 analyzes the explanatory power of the proposed prediction model based on feature importance and the Shapley additive explanations (SHAP) method, from the perspective of the time series features of building energy consumption prediction. Finally, the proposed model was proved effective through experiments.

## 2. Prediction Principle of Building Energy Consumption

In traditional prediction models of building energy consumption, an information loss may occur due to the connection vector between the encoder and the decoder. To solve the problem, this paper introduces the TPAM to the existing prediction framework. The new prediction model can make better predictions of building energy consumption, during the handling of the input time series, which involve multiple variables.  Figure 1 illustrates the architecture of the TPAM-based prediction model for building energy consumption.

Compared with traditional attention mechanism, the TPAM can effectively handle the multivariate input time series for the forecast of building energy consumption. This mechanism can mine more deep-seated information from the multivariate input time series, according to the weights of specific variables, and the acquired local features. It can also identify the lost position and other key information. The TPAM mainly encompasses two parts: a time detection module of convolutional neural network (CNN) and an attention weighting module. The workflow of the TPAM is as follows:

In the prediction model, the bidirectional gated recurrent unit (BiGRU) layer mainly computes the n-dimensional hidden state *f*_*i*_ of each time step, and then derive the hidden state matrix *F* = {*f*_*e *−* q*_, *f*_*e*-* *+* *1_,…, *f*_*e *−* *1_}, where *q* is the length of the sliding window. For the time series for building energy prediction, the states of each variable at all time steps can be represented by a row vector of the hidden state matrix E. The states of all variables at each time step can be characterized by a column vector in that matrix. Then, a one-dimensional (1D) CNN can be called to extract the variable time pattern:

(1) $$\begin{array}{c} F_{i,j}^{D}=\sum_{k=1}^{q}F_{i,\left(e-q-1+k\right)}\times D_{j,E-q+k}. \end{array}$$

Formula (1) performs a convolution operation *D* with *l* filters and the kernel size of 1 × *E* over the row vector of *F*, producing the time pattern matrix *F*^*D*^ corresponding to that variable. Let *F*_*ij*_^*D*^ be the calculation result of the *i*-th row vector and the *j*-th kernel; *F*_*i*_^*D*^ be the *i*-th row of matrix *F*^*D*^; *Q*_*x*_ be the trainable weight matrix; *f*_*e*_ be the hidden state outputted by the BiGRU layer. Then, the variable time pattern can be evaluated by the following:

(2) $$\begin{array}{c} g\left(F_{i}^{D},f_{e}\right)={\left(F_{i}^{D}\right)}^{E}Q_{x}f_{e}. \end{array}$$

To obtain multiple variables that facilitate the prediction of building energy consumption, the TPAM would determine the attention weights by sigmoid function. The attention weight *β*_*i*_ can be calculated by the following:

(3) $$\begin{array}{c} \beta_{i}=\text{sigmoid}\left(g\left(F_{i}^{D},f_{e}\right.\right). \end{array}$$

Finally, the context vector vtue can be obtained as the weighted sum of the vectors in row *F*^*D*^:6

(4) $$\begin{array}{c} u_{e}=\sum_{i=1}^{n}\beta_{i}F_{i}^{D}. \end{array}$$

The GA optimization of the BP neural network intends to improve the initial weights and thresholds of the network. However, the traditional GA has difficulty in optimizing the structural parameters of the neural network. The main difficulty lies in the variation of chromosome length with the number of hidden layers. To solve this problem, the GA is improved in this research. In the improved GA, the single-point crossover is adopted as follows:

(5) $$\begin{array}{c} {\tilde{a}}_{1,j}\left(e\right)=0.5\times \left[\left(1+\Phi_{j}\right)a_{1j}\left(e\right)+\left(1+\Phi_{j}\right)a_{2j}\left(e\right)\right],\\ {\tilde{a}}_{2,j}\left(e\right)=0.5\times \left[\left(1+\Phi_{j}\right)a_{1j}\left(e\right)+\left(1+\Phi_{j}\right)a_{2j}\left(e\right)\right], \end{array}$$

where

(6) $$\begin{array}{c} \Phi_{j}=\left\{\begin{array}{cc} {\left(2\lambda_{j}\right)}^{1/\gamma +1}\text{,} & \text{if}\lambda_{j}\leq 0.5,\\ {\left(\frac{1}{2\left(1-\lambda_{j}\right)}\right)}^{1/\gamma +1}, & \text{Otherwise},\lambda_{j}\in V\left(0,1\right)\text{with}\lambda >0\text{being the dispersion index}. \end{array}\right. \end{array}$$

The improved GA adopts polynomial mutation. Suppose the mutation operator is *u*_*l*_′=*u*_*l*_+*ξ* · (*v*_*l*_ − *k*_*l*_), *ξ*_1_=(*u*_*l*_ − *k*_*l*_)/(*v*_*l*_ − *k*_*l*_), and *ξ*_2_=(*v*_*l*_ − *u*_*l*_)/*v*_*l*_ − *k*_*l*_. Let *v*denote a random variable in [0, 1]; *γ*_*n*_ denote the dispersion index; *u*_*l*_ denote a parent individual. Then, *ξ* can be calculated by the following:

(7) $$\begin{array}{c} \xi =\left\{\begin{array}{cc} {\left[2v+\left(1-2v\right){\left(1-\xi_{1}\right)}^{\gamma_{n}+1}\right]}^{1/\gamma_{n}+1}-1, & \text{if}v\leq 0.5,\\ 1-{\left[2\left(1-v\right)+2\left(v-0.5\right){\left(1-\gamma_{2}\right)}^{\gamma_{n}+1}\right]}^{1/\gamma_{n}+1}, & \text{if}v>0.5. \end{array}\right. \end{array}$$

## 3. Construction of the Energy Consumption Prediction Model

The TPAM-based energy consumption prediction model consists of three parts: BiGRU encoder, TPAM, and BiGRU decoder.  Figure 2 illustrates the input of the TPAM. The prediction model is executed in the following steps:

**Step 1 .**

Let *a*_*e*_ be the input time series at the current time step; *f*_*e − *1_ be the hidden state at the previous time step; *f*_*e*_ be the hidden state at the current time step *e*. After importing *a*_*e*_, and *f*_*e − *1_ into the encoder, *f*_*e*_ can be calculated by the following:

(8) $$\begin{array}{c} f_{e}={\text{BiGRU}}_{\text{encoder}}\left(a_{e},f_{e-1}\right). \end{array}$$

**Step 2 .**

Let *b*_*e − *1_ be the previous output series; *r*_*e − *1_ be the hidden state of the previous time step; *r*_*e*_ be the hidden state of the current time step. Based on *b*_*e − *1_ and *r*_*e − *1_, the decoder can compute *r*_*e*_:

(9) $$\begin{array}{c} r_{e}={\text{BiGRU}}_{\text{decoder}}\left(b_{e-1},r_{e-1}\right). \end{array}$$

**Step 3 .**

Let *Q*_*u*_ be the parameter matrix. The context vectors *u*_*e*_ and *r*_*e*_ can be connected to obtain the following:

(10) $$\begin{array}{c} {\hat{r}}_{e}=\tanh\left(Q_{u}\left[u_{e};r_{e}\right]\right). \end{array}$$

**Step 4 .**

Let *Q*_*r*_ be the parameter matrix. Then, *b*_*e*_ can be solved based on the SoftMax function:

(11) $$\begin{array}{c} b_{e}=\text{softmax}\left(Q_{r}{\hat{r}}_{e}\right). \end{array}$$

The energy consumption of buildings is affected by various factors. The time series inputted to predict building energy consumption can be divided into the historical energy consumptions at the *n* previous moments, time variables, and weather variables. Here, the objective function of building energy consumption prediction is defined as follows:

(12) $$\begin{array}{c} \hat{b}=G\left(A,B\right), \end{array}$$

where *A*=(*PE*, *SF*, *XO*, *QR*, *F*, *C*, *Q*, *N*, *W*), with *PE*, *SF*, *XO*, *QR*, *F*, *C*, *Q*, *N*, and *W* being the various input variables, such as wind velocity, humidity, temperature, and sun intensity. The historical energy consumptions at the *n* previous moments are denoted by *B* = (*K*_*e*_, *K*_*e − *1_, *K*_*e − *2_, *K*_*e − *3_, *K*_*e − *4_,…, *K*_*e − n*_), with *n* being the window length of the historical data. The predicted values for the *m* future moments are denoted as *b*^*∗*^=(*b*_*e*+1_*∗*, *b*_*e*+2_*∗*, *b*_*e*+3_*∗*,…, *b*_*e*+*m*_*∗*).  Figure 3 illustrates the input data of the model.

The Adam algorithm can dynamically adjust the learning rate of each parameter, making the update of parameters steadier. In actual applications, this algorithm outshines most gradient-based optimizes. This paper relies on the Adam algorithm to iteratively update the weight and bias of each node of the prediction model, in order to obtain an adaptive learning rate. Let *n*_*e*_ and *m*_*e*_ be the estimation for the first-order moment of gradients, and that for the second-order moment of gradients; *n*_*e*_′ and *m*_*e*_′ be the correction for *n*_*e*_ and *m*_*e*_, respectively; *γ* be the learning rate. Then, we have as follows:

(13) $$\begin{array}{c} n_{e}=\lambda *n_{e-1}+\left(1-\lambda \right)*h_{e},\\ m_{e}=u*m_{e-1}+\left(1-u\right)*h_{e}^{2},\\ \Delta \omega_{e}=-\frac{{\hat{n}}_{e}}{\sqrt{{\hat{m}}_{e}}+\sigma }*\gamma , \end{array}$$

where *n*_*e*_′ and *m*_*e*_′ can be viewed as unbiased estimates of expectations. The loss function of the model is the easily solvable mean squared error (MSE):

(14) $$\begin{array}{c} MSE=\frac{\sum_{i=1}^{m}{\left({\hat{b}}_{i}-b_{i}^{o}\right)}^{2}}{m}, \end{array}$$

where *m* is the number of samples; *b*_*i*_ and *b*_*i*_^*o*^ are actual value and predicted value, respectively.

## 4. Analysis on Explanatory Power

Based on feature importance and the SHAP method, the explanatory power of the proposed prediction model was analyzed, from the perspective of the time series features of building energy consumption prediction.

To disturb each time series for predicting building energy consumption, noises are added to the eigenvalues of each time series. The model performance is measured by MSE (14). The importance of feature *l* can be calculated by the following:

(15) $$\begin{array}{c} \Delta_{l}=\left|MSE_{li}-MSE_{lj}\right|. \end{array}$$

Let MSE_*i*_ and MSE_*j*_ denote the MSE of the model before and after noise addition, respectively. The greater the SHAP feature importance, the more important the features of a time series. The SHAP feature importance can be calculated by the following:

(16) $$\begin{array}{c} GY_{j}=\frac{1}{m}\sum_{i=1}^{m}\left|\Psi_{j}^{\left(i\right)}\right|, \end{array}$$

where *m* is the sample size; Ψ_*j*_^(*i*)^ is the Shapley value of the *j*-th feature in the *i*-th time series sample.

The interaction effect between time series features can be measured by the effect of the combinatory features added to a single time series feature. The Shapley interaction index of two time series features can be defined as follows:

(17) $$\begin{array}{c} \Psi_{i,j}=\sum_{r\subseteq \left\{a_{1},...,a_{o}\right\}/\left.\left\{a_{i},a_{j}\right\}\right\}}\frac{\left|R\right|!\left(o-\left|R\right|-2\right)!}{2\left(o-1\right)!}\xi_{ij}\left(R\right). \end{array}$$

If *i*≠*j*, we have the following:

(18) $$\begin{array}{c} \xi_{ij}\left(R\right)=g\left(R\cup \left\{a_{i},a_{j}\right\}\right)-g\left(R\cup \left\{a_{i}\right\}\right)-g\left(R\cup \left\{a_{j}\right\}\right)+g\left(R\right). \end{array}$$

## 5. Experiments and Result Analysis

To highlight the universality of predicting building energy consumption, two different public datasets were selected from China and a foreign country for our experiments.

Out of the various factors affecting building energy consumption, the change of the local climate is a leading factor. This paper summarizes the energy consumption of target buildings at different temperatures. The results in Figure 4 show that when the temperature is below 20°C, the mean energy consumption of buildings does not change significantly with the rise of the mean temperature; when the temperature is above 20°C, the mean energy consumption of buildings surges up with the growth of the mean temperature, mainly due to the increase of refrigeration loads.

To demonstrate its effectiveness, the proposed prediction model of building energy consumption was compared with recurrent neural network (RNN) (model 1), GRU (model 2), LSTM (model 3), deep *Q* network (DQN) (model 4), and dueling DQN (model 5).  Figure 5 compares the prediction results of the different models. It can be observed that the prediction of our model is closer to the actual value, and more accurate than that of other models. Besides, the prediction effect of our model is better, when the refrigeration load consumes much energy during the working period, as evidenced by the minimum prediction error.

Table 1 compares the prediction errors of different models. Obviously, the five models differed significantly in the prediction accuracy on the time series for building energy consumption. Our experiment lasted five months. The results show that our model had a 3–6% lower MAPE and 35–50% lower MSE than the other models. The low MAPE and MSE demonstrate the good generalization and robustness of our model.

As a tool for explaining the prediction of building energy consumption, SHAP can explain the quality of the prediction on a single test sample, and the importance of complex time series features.  Figure 6 compares the metrics of different models. It can be seen that our model predicted building energy consumption better than the other models, as evidenced by its superior fitting effect on the time series for building energy consumption.

Table 2 presents the SHAP values of the features of the 11 variables below the mean prediction output. The SHAP values of variables PE, QR, *C*, *Q*, and N were smaller than zero, indicating that these variables negatively affect the prediction output of our model. The SHAP values of the other variables are greater than zero, suggesting that they promote the prediction output of our model. In the meantime, the positive effect of the eigenvalues corresponding to the 11 features was smaller than the negative effect of these eigenvalues. Thus, the output of the time series for building energy consumption is smaller than the mean prediction output.

Figure 7 shows the importance of the SHAP features of the 11 variables. It can be observed that the high-ranking variables exert a significant impact on the prediction output of building energy consumption. Among them, the SHAP feature corresponding to *b*^*∗*^ was the most important, indicating that *b*^*∗*^ contributes the greatest to the output of the energy consumption prediction model. By contrast, the SHAP feature corresponding to wind velocity PE was the least important, indicating that PE contributes the least to the output.

## 6. Conclusions

This paper optimizes the explanatory power of the prediction model for building energy consumption. Specifically, the authors displayed the architecture of the TPAM-based prediction model for building energy consumption and introduced the principle of predicting building energy consumption. Then, they went on to illustrate the input of the TPAM and explain the execution steps of the model. Based on feature importance and SHAP method, the explanatory power of the proposed prediction model was analyzed, from the perspective of the time series features of building energy consumption prediction. Through experiments, this paper summarizes the energy consumption of target buildings at different temperatures and identifies the main reasons for the influence of temperature on building energy consumption. To demonstrate its effectiveness, our prediction model for building energy consumption was compared with different models. The comparison of prediction errors proves the effectiveness of our model. In addition, the authors displayed the SHAP values of the features of the 11 variables below the mean prediction output and exhibited the importance of the SHAP features of these variables. Finally, the explanatory power of our model was analyzed.

Due to the limited data volume, it is difficult to build an energy consumption prediction model for each season. In future, as more data become available, the research of building energy prediction model will be further improved and better prediction effect will be realized.

## Figures and Tables

**Figure 1:** TPAM-based prediction model for building energy consumption.

**Figure 2:** Input of TPAM.

**Figure 3:** Input data of the model.

**Figure 4:** Influence of temperature on building energy consumption.

**Figure 5:** Prediction results of different models.

**Figure 6:** Metrics of different models. RMSE and MAE are short for root mean square error and mean absolute error.

**Figure 7:** Importance of the SHAP features of the 11 variables.

**Table 1:** Prediction errors of different models.

Period	Metric	Dataset					
		Model 1	Model 2	Model 3	Model 4	Model 5	Our model
January	MAPE	16.24%	14.73%	12.15%	10.58%	13.96%	6.48%
	MSE	7.19	6.33	5.24	4.35	3.85	2.39

February	MAPE	17.54%	15.21%	14.62%	9.58%	9.16%	5.37%
	MSE	7.98	6.08	5.03	4.81	4.59	2.74

March	MAPE	16.61%	14.73%	12.54%	9.38%	14.71%	6.85%
	MSE	7.49	6.63	5.06	4.71	4.38	2.74

April	MAPE	17.28%	16.11%	13.62%	11.48%	9.62%	5.37%
	MSE	6.99	6.52	6.09	4.35	4.18	2.63

May	MAPE	17.84%	17.03%	16.95%	11.41%	13.64%	6.17%
	MSE	7.84	5.87	5.16	4.95	4.35	2.81

Mean	MAPE	15.78%	114.57%	13.05%	11.62%	13.84%	6.37%

MAPE is short for mean absolute percentage error.

**Table 2:** SHAP values of the features of the variables below the mean prediction output.

Variable	Eigen value	SHAP value	Variable	Eigen value	SHAP value
PE	43	−5.1273	*C*	10	−0.4627
SF	42.8	1.6259	*Q*	75.69	−0.3162
XO	189	2.4815	*N*	184.53	−1.4851
QR	40.53	−2.4183	*W*	78	0.4195
*F*	72	0.7481	*B*	15	0.3268
*b* ^*∗*^	36	0.1245			

## Data Availability

The data used to support the findings of this study are available from the corresponding author upon request.

## References

[1] Yang X., Zhang S., Xu W. (2019). Impact of zero energy buildings on medium-to-long term building energy consumption in China. *Energy Policy*.

[2] Zhang M., Ge X., Zhao Y., Xia-Bauer C. (2019). Creating statistics for China’s building energy consumption using an adapted energy balance sheet. *Energies*.

[3] Huang Z., Ge J., Zhao K., Shen J. (2019). Post-evaluation of energy consumption of the green retrofit building. *Energy Procedia*.

[4] Wang Y., Wang P. (2022). Effects of building physics form on energy consumption for buildings. *Journal of Physics: Conference Series*.

[5] Ji C., Hong T., Kim H., Yeom S. (2022). Effect of building energy efficiency certificate on reducing energy consumption of non-residential buildings in South Korea. *Energy and Buildings*.

[6] Wenninger S., Kaymakci C., Wiethe C. (2022). Explainable long-term building energy consumption prediction using QLattice. *Applied Energy*.

[7] Touzani S., Ravache B., Crowe E., Granderson J. (2019). Statistical change detection of building energy consumption: applications to savings estimation. *Energy and Buildings*.

[8] Li H. J., Qiao Z., Chen W., Zeng X. Q., Wu L. (2019). Research on public building energy consumption prediction method based on NAR neural network prediction technology. *E3S Web of Conferences*.

[9] Tian C., Li C., Zhang G., Lv Y. (2019). Data driven parallel prediction of building energy consumption using generative adversarial nets. *Energy and Buildings*.

[10] Xie Q., Ni J. Q., Bao J., Su Z. (2019). A thermal environmental model for indoor air temperature prediction and energy consumption in pig building. *Building and Environment*.

[11] Sha G., Qian Q. Prediction of commercial building lighting energy consumption based on EPSO-BP.

[12] Li C., Ding Z., Yi J., Lv Y., Zhang G. (2018). Deep belief network based hybrid model for building energy consumption prediction. *Energies*.

[13] Chen S., Ren T. T., Wu Z. C. (2018). Research on neural network optimization algorithm for building energy consumption prediction. *Journal of Computational Methods in Science and Engineering*.

[14] Ahmad M. W., Mourshed M., Rezgui Y. (2017). Trees vs Neurons: comparison between random forest and ANN for high-resolution prediction of building energy consumption. *Energy and Buildings*.

[15] El-Gohary K., El-Gohary N. (2016). Building lighting energy consumption prediction for supporting energy data analytics. *Procedia Engineering*.

[16] Son H., Kim C., Kim C., Kang Y. (2015). Prediction of government-owned building energy consumption based on an RReliefF and support vector machine model. *Journal of Civil Engineering and Management*.

[17] Ullah I., Ahmad R., Kim D. (2018). A prediction mechanism of energy consumption in residential buildings using hidden Markov model. *Energies*.

[18] Kim S., Kim D. (2018). Prediction-learning algorithm for efficient energy consumption in smart buildings based on particle regeneration and velocity boost in particle swarm optimization neural networks. *Energies*.

[19] Mena R., Rodríguez F., Castilla M., Arahal M. R. (2014). A prediction model based on neural networks for the energy consumption of a bioclimatic building. *Energy and Buildings*.

[20] Zhang Y., Chen Q. Prediction of building energy consumption based on PSO-RBF neural network.

[21] Ferlito S., Atrigna M., Graditi G. (2015). Predictive models for building’s energy consumption: an Artificial Neural Network (ANN) approach. *Xviii Aisem Annual Conference*.

[22] Yin R., Yin J. (2022). Prediction method of energy consumption for high building based on LMBP neural network. *Energy Reports*.

[23] Jing W., Zhen M., Guan H., Luo W., Liu X. (2022). A prediction model for building energy consumption in a shopping mall based on Chaos theory. *Energy Reports*.

[24] Li X., Liu S., Zhao L., Meng X., Fang Y. (2022). An integrated building energy performance evaluation method: from parametric modeling to GA-NN based energy consumption prediction modeling. *Journal of Building Engineering*.

[25] Chou I., Chou S. Y. (2022). A hybrid RF-LSTM based on CEEMDAN for improving the accuracy of building energy consumption prediction. *Energy and Buildings*.

